# The Kawa Model: A Self-Reflection Tool for Occupational Therapy Student Development in Practice Placements in Australia

**DOI:** 10.1155/2023/2768898

**Published:** 2023-01-12

**Authors:** Ornissa Naidoo, Chantal Christopher, Thanalutchmy Lingah, Monica Moran

**Affiliations:** ^1^Western Australia Country Health Service-Midwest, Geraldton, Western Australia 6530, Australia; ^2^Western Australia Centre for Rural Health, Geraldton, Western Australia 6530, Australia; ^3^School of Allied Health, University of Western Australia, Perth, Western Australia 6009, Australia; ^4^School of Health Sciences, University of Kwa Zulu Natal, University Road, Westville Private Bag X 54001, Durban 4000, South Africa

## Abstract

**Introduction:**

The Kawa Model is a conceptual occupational therapy model of practice that uses the metaphor of a river as a medium to support the exploration of self, life events, and environment. In this study, the Kawa Model was used by occupational therapy students during a practice placement in a remote community setting as a tool to support learning, build self-awareness, and promote reflection on personal and professional development.

**Method:**

The study used an exploratory qualitative research design. Six student participants were purposively recruited and orientated to the use of the Kawa Model at the beginning and throughout their remote community practice placement. Semistructured interviews were used to collect data which were analysed thematically using interpretative phenomenological analysis (IPA). *Findings*. Analysis of the student transcripts revealed three overarching themes: self-awareness, the development of personal and professional skills, and working with metaphor. All students identified the model as a reflective tool that enhanced their understanding of their student selves in a remote setting. The students described the growth of various professional skills including communication, goal planning, and confidence. Whilst initially students found the metaphor challenging to fathom, throughout their placement, they found it impactful for comprehending their development of self.

**Conclusion:**

This study revealed that the students' self-awareness and personal and professional development were influenced by their engagement with and application of the Kawa Model. Repeated engagement with the Kawa Model enhanced the students' journey of personal and professional skill development.

## 1. Introduction

In 2006, Iwama et al. [1] presented a new conceptual occupational therapy practice model designed around a metaphor that challenged the dominant cultural constructs of the profession. It is widely acknowledged that modern-day occupational therapy evolved within a Western epistemology. Contemporary criticism of the profession has been its tethering to western values and perspectives, including the constructs of individuality, independence, and productivity. Hammell [2] discusses how this potentially excludes communities that do not ascribe to those values. In contrast, the Kawa Model is a dynamic occupational therapy model informed by Eastern philosophy. It positions individuals as integral aspects of a collective ecological whole and aims for a more inclusive representation of the human experience [3]. Within the Kawa (River) Model, the river represents a metaphor for life, where a deep, freely flowing river characterises well-being and the chronological experience of life. Well-being (the flow of the river) is affected by the environment (represented by the river walls and riverbed), life circumstances (represented by rocks in the river), and assets and liabilities (represented by driftwood). The self is seen as a whole entirety that is deeply connected with society and circumstances [1]. Thus, in the Kawa Model, the “self” which may be seen as the river flow, is shaped by the environment (rocks) and societal constructs (driftwood).

The use of metaphors in occupational therapy practice has a long history. The profession's founders in 1915 used the metaphor of “a new pathway” to describe the experience of clients when engaging in new activities to promote well-being [4]. Mallinson et al. [5], in 1996, described metaphors used by clients to explain their experiences of illness, disability, and impairment. Metaphors are also commonly used in health professions education to introduce students to complex concepts, such as bridging the theory-practice divide [6].

The Kawa Model has been researched predominantly in clinical settings [7–13]. In addition, the model has been implemented with a diversity of people including parents of autistic children where a modified model found that the experiences/goals of the parents were intertwined with that of their children. This is in keeping with the social and environmental constructs of the model which states that the life flow of an individual is linked to the walls and beds of a river [14]. In another study, the Kawa Model was used together with other tools, to try and elicit Indigenous Australians' perspectives of health and physical activity. Participants were offered to draw or paint their “river” as a means to depict their life and views on what enabled or complicated their ability to be “active/healthy” [15]. A recent scoping review summarised a range of settings in which the Kawa Model was used. Our study extends the evidence for using the Kawa Model in the education space within a rural environment [13].

Iwama et al. proposed that the model can increase therapists' awareness of their cultural lens and help them understand the culturally nuanced nature of their occupational practice [1]. Related to this, there is an emerging body of knowledge regarding the application of the Kawa Model in nonclinical settings such as education, professional development, and professional collaboration in the workplace [13, 16–19]. In the professional education sphere, Tripathi and Middleton [18] described the use of the Kawa Model with occupational therapy students to plan, implement, measure, and provide future recommendations on their professional development. Smith [17] used the Kawa Model with occupational therapy students to identify students' barriers to learning, personal attributes, and circumstances and the environment that impacted their course learning. Smith suggests that by using the model as a tool for their development, the students appreciated its use in practice [17]. The Kawa Model has also been used as a reflective tool for learning in final-year student placement [20]. In this study, the Kawa Model is proposed as a reflective learning resource to support occupational therapy students completing their practice placement in a remote location in Western Australia.

There is a growing concern in the health and education literature that students are almost universally educated in urban settings and their preparation for professional placement is “placeless” and disjoined from the place in which it will be enacted [21]. This generates increased requirements for rural and remote educators to equip students with knowledge and skills to adapt to nonmetropolitan placements. Introducing resources for learning and practice such as the Kawa Model purports to have universal application and reflect metaphorical elements that align with practice-placement sites may support students to engage dynamically in their learning placements. The student, by using the Kawa Model across various settings, could expand their knowledge of their “river flow” across a variety of contexts and amidst various cultures.

## 2. Purpose of Study

The purpose of this study was to explore students' perceptions and experiences of applying the Kawa Model to themselves in rural community placements and to explore how the model may contribute to developing personal and professional practice skills.

## 3. Method

Ethical approval for this study was provided by the University of Western Australia (RA/4/20/4960). Pseudonyms are used to maintain the anonymity of the students who participated in the study. An exploratory qualitative research design method was used.

### 3.1. Context

This study was carried out in a remote location in the Pilbara region in Western Australia, 1500 km from the closest major city. This arid region is rich in natural mineral resources and is characterised by a very low-population density of less than one person per kilometre [22]. The Pilbara has a rich indigenous cultural heritage, with local aboriginal groups making up about 25% of the population. Occupational therapy students travel from metropolitan universities around Australia to gain experience in this remote location. All students were accommodated by the University Department of Rural Health in the Pilbara and were supervised by the same occupational therapy practice educator during their eight-week placement. Their practice-placement sites included aboriginal playgroups, primary schools, an aboriginal-aged care facility, and an aboriginal home and community centre.

### 3.2. Sampling

Purposive sampling was used to recruit occupational therapy students in their fourth and final year of study. Six students in three pairs consented to participation in the study in the 2019 academic year. The students had varying levels of knowledge and experience in using the Kawa Model, with most reporting minimal prior experience in its application. All students were female, between the ages of 20 and 30 years. Students came from universities in Western Australia and Queensland, another state in Australia. There are no universities in the Pilbara. Demographics of the sample is shown in Table 1.

### 3.3. Procedure

Students attended placement in pairs. Over 2019, three pairs (six) of occupational therapy students on placement in the Pilbara were informed about the study by an administrative officer not connected with the study, and all agreed to participate. The students attended a training session with the occupational therapy practice educator that included an introduction to the Kawa Model and readings about its application in various clinical, nonclinical, and professional practice settings. The training was piloted on six other students before the research process.

During the training, the students had an opportunity to practice applying the model on themselves and with their paired peers using guided templates and illustrations (see Figure 1). This training session involved students taking a cross-section of their river at the start of their placement to explore the various elements of their personal Kawa and its impact on their river flow. The students then examined their cross-section of the river, analysing options to reduce boulders, and perhaps use their driftwood to enhance their river flow (see Figure 2). In this way, they worked with their peer (facilitators) to set personal and professional goals. Each student took a turn as a facilitator and as a subject in the training session to complete the cross-section of the river, and then develop their goals.

This learning session was informed by Kolb's experiential learning cycle [23] and Morris' revision of the model where the rural context is emphasised as contributing to the “contextually rich” concrete experience [24]. Similar to Morris' revision, students on the remote placement were active participants, using experiential learning and critical reflection to make meaning of the training within the rural context.

Students were encouraged by their practice educator to use and repeat the Kawa Model process throughout their placement either with their peers or alone, to monitor their river/life flow. During weekly individual supervision, the practice educator encouraged discussion of the use of the Kawa Model process as a self-directed learning tool. Similar sessions used the Kawa Model process at both the halfway mark and at the end of the practice placement with all student pairs.

### 3.4. Data Collection

A semistructured interview guide was developed collaboratively by the research team of four experienced occupational therapy educators (see Table 2). The interview focused on exploring the students' experiences of using the Kawa Model process on themselves during their placement. All six students were individually interviewed at the end of their placements by the same member of the research team who was located in another part of the state and who had not been involved in their placement planning, coordination, supervision, or assessment. Information and consent forms were distributed to the students by the administration officer not involved in the study. Written consent was obtained from each student to participate in the research and to record their interview. The interviews were completed via a video conferencing platform (Zoom) and recorded using a digital recorder. The recording function on Zoom was not used to maintain the anonymity of the students. The interview duration ranged from 20 minutes to 45 minutes. Digital interview files were transcribed by a professional transcription service. In line with ethical requirements, all digital and text files were stored in a password-protected electronic folder on the University of Western Australia server. Only members of the research team had access to this folder.

### 3.5. Data Analysis

Interpretative phenomenological analysis (IPA) is a research approach that allows researchers to capture the qualitative and experiential aspects of the human experience and helps examine how people make sense of their life experiences [24].

IPA utilises an experiential method to explore the human experience from the point of view of those who are having the experience [25]. The IPA process supports researchers to uncover meanings through the interpretation of qualitative data whilst acknowledging that those interpretations are always generated through the lens of the previous experiences of the participant and of the researcher. The interpretative phenomenological analysis supports an idiographic exploration of each case so that the diversity of experiences of individuals can be uncovered. The research team followed the analysis process outlined by Smith et al. [26] which is described in Table 3. In addition, the team met fortnightly to reflect on the analysis process and maintained detailed recordings of their ideas, reflections, and emerging interpretations throughout the project.

The analysis and trustworthiness of the findings were strengthened by the four researchers meeting fortnightly after independently analysing the transcripts and comparing their impressions until a final consensus was reached. A detailed document trail was kept by the primary investigator through reflective notes of her own experiences and involvement in the research process. The reflective notes were kept to support analysis and interpretation and stored on a secure research drive.

## 4. Findings

Analysis of the transcripts elicited three overarching themes: theme 1: self-awareness, theme 2: personal and professional development skills, and theme 3: working with the metaphor.

Theme 1 describes how engaging with the Kawa Model process helped students become more self-aware which further enabled their identification and setting of appropriate goals for personal and professional skill development seen in theme 2. Theme 3 relates to the students' experiences of interacting with the metaphor, their struggles, and their evolving understanding of the metaphor and themselves.

In the following sections, each theme is described in detail. Verbatim student quotations from the data transcripts are selectively tabulated to evidence the subthemes (Tables 4–6). Following each table, the themes and subthemes are explored further, with additional evidence from the study.

### 4.1. Theme 1: Self-Awareness

This theme describes the students' development of self-awareness through self-reflection, self-understanding, self-evaluation, and self-motivation. All students reported that using the Kawa Model process enhanced their river flow (described in Section 3.3) through their understanding of themselves as illustrated in the quotes.

Students reported that applying the Kawa Model process facilitated a metacognitive framing through checking in and reflecting on themselves and the progress they were making in their placement (Quotes 1.1.1 and 1.1.2). The students who described themselves as being reflective reported that the experience of drawing their Kawa enhanced their skills in self-reflection. They were able to visually interpret the drawings concerning themselves and deepen their self-understanding (Quote 1.2). This visual processing also enhanced students' self-evaluation related to their self-belief or self-doubt (Quote 1.3).

The iterative-structured process of engaging with the model for the students' practice placement created an opportunity for self-awareness and thereby enhanced their journey of learning and professional development over time. The process and frequency of use of the model motivated the students to evaluate the efforts they were making and redirect their learning. Ava, in Quote 1.4, suggests that whilst you might not complete the tool comprehensively every week, she believes that the Kawa Model is a good “tool” to use on student placement weekly. Overall, students perceived that repeating the Kawa Model process provided opportunities to enhance their self-awareness and self-confidence.

Whilst describing the Kawa Model process, Kylie also elaborates on one of her boulders being her “lack of confidence,” and how this boulder influenced her river flow and eventually became smaller. “I think one of my boulders was (lack of) confidence. At the start of this placement, it was very big. And that is just generally …I see that happens all the time. But during my time redoing my Kawa, I noticed that it is not such a big impact anymore” Kylie.

The visual nature (Quote 1.3) of the Kawa Model allowed the students to objectively evaluate their river flow by exploring the Kawa elements such as the size of the boulders (barriers to learning) they were experiencing and how they changed throughout their placement. It is through the visual nature and the process that awakened Ella to the realisation that she had increased her confidence (Quote 1.5).

Although the students identified the benefits of using the model as a reflective tool, there were mixed responses on whether they would use the model in the future. One student who saw herself as not being reflective, found the Kawa Model challenging to start with and later felt “it was really helpful and effective for my planning and my placement as well. “It improved my self-awareness in that I had never actually broken it down to think about it” Mia. Even though she found the model effective, she revealed that she would still require prompts to reflect in the future.

“I do not know if I would use the Kawa on myself again purely because I am not someone who self-reflects a lot,…unless prompted.” Mia

Some self-declared reflective students reported that they would use the Kawa Model process on themselves again, or in their service team. Other students reported that they would reengage with the model if they were having a particularly challenging time in their future lives.

“If I was having a real rough time in my life, I would use the Kawa, and that is even to just deal with stress at work or just generally in my life while I am working. It depends on where I would use the Kawa for the situation.” Kylie

### 4.2. Theme 2: Personal and Professional Skill Development

This theme explores the students' perceptions of how the application of the Kawa Model process provided them with opportunities to develop their personal and professional skills. The table illustrates the subthemes related to this and the verbatim quotes.

Participants reflected that applying the Kawa Model to themselves helped to consolidate their understanding of the model, acknowledge the theory-practice relationship, and built their confidence in using the model with clients (Quote 2.1.).

Working on one's own Kawa Model process provided the students with the opportunity to explore the significance of the components of the river as well as the river flow (Quote 2.1). Thus, they could “hone-in” and identify personal and professional development (life) that they needed to work on (Quote 2.2).

The iterative process of completing the Kawa process throughout their placement assisted the students to identify new practical skill areas (Quote 2.2); apply this knowledge to set realistic goals for their learning (Quote 2.3) and compare and review progress over time (Quote 1.3). Amelia described this iterative process of reviewing her goals.

“We would bring our previous Kawa to the Kawa session, and we did a very quick comparison to see which boulders had shrunk or any new boulders, and it revealed that within the week, we had worked on the goals that we set in the previous Kawa session.” Amelia

Recalling her work with a peer, Amelia commented on the effect of the process on their mutual understanding and evolving relationship.

“With my colleague, we looked at both our Kawas and made goals for how to improve our communication. We did not write them down, but we were more aware of what we were both working on so that our relationship worked better…. So, it was a nice getting to know each other kind of activity…. I guess because we were open straightaway; the whole process worked quite well for the following weeks of placement.” Amelia

Most of the students reported that working with a peer provided them with an opportunity for self-disclosure early in the peer-relationship collaboration, which facilitated understanding of the other, deepened their communication, and facilitated opportunities for peer-assisted learning.

“Yeah, so it was good to practice with her as well, and she really enjoyed doing it for herself.” Grace

“Having a peer (she) provided some perspective of seeing, like, ‘Oh no, we have not like minimised that rock from the last time.'” Amelia

One student reflected that some students might find working in pairs confronting if they did not know their peers “individuals can have certain areas that they do not want to bring up to someone that they have just met” (Kylie). For this reason, students had the option to implement the Kawa Model on their own if they felt more comfortable.

Some students introduced modifications or suggestions on how the Kawa Model could be used to better support their learning both during and outside of supervision meetings. Amelia suggested that the supervisor further prompt her on using the Kawa Model and to “map it out in a Kawa,” as she sometimes “got lazy with the frequency of use.”

Ava suggested that we could also change the cross-section to specific times of life, allowing the focus to change. This would allow one to concentrate on specific areas to enhance.

“…so it can be a general one and then other times you could specify that you are going to focus on what the boulders are in a particular relationship or regarding a particular assignment. And I think that can also help you hone-in because you are now looking at a smaller area of your life, and so, you have to identify all the boulders, and that assists to help you in that specific area.” Ava

As students became more familiar and confident with the model, they took opportunities to teach one another and to share the model with other students who attended peer-assisted learning (PAL) sessions with them online from other practice-placement locations.

“The other student (OT student on a different placement) was teaching us because she had more experience about assessments and different experiences and knowledge. We always thought that we were not really bringing much to her, but we did bring the Kawa Model which was good, so we showed her that. She really enjoyed drawing it. I think as OTs, a lot of us are quite visual learners. Yeah, so it was good to practice with her.” Grace

The quotes above describe students' perceptions of their development of personal and professional skills including self-confidence and peer and team communication, as well as formulation of goals.

### 4.3. Theme 3: Working with the Metaphor

There is some evidence in the literature regarding clients' responses to the metaphor embedded within the Kawa Model [7–13, 15]. There is limited published information, however, regarding occupational therapy students' responses to the metaphor. Even though most of the students in this study had some exposure to the Kawa at university and all received training at the start of their placement, they reported difficulty in understanding and applying the metaphor early in their placement. Some of these challenges are exposed in this theme. Over time, students immersed themselves in the model and reported a deeper understanding of the metaphor's visual and figurative elements.

The Kawa Model utilises the universal metaphor of a river to generate descriptions of life from the user's perspective. Using the Kawa Model, it required the student to understand the inherent conceptualisation (within the metaphor), and then to apply the metaphor in the unpacking of either their own or their peer's life experiences. As the metaphor is read through an individual lens by the students and their peers, it is loaded with contextual interpretations. Working with metaphor provided both challenges and meaningful experiences for students, particularly those who were not familiar with the model before their placement. Students reported that they initially found it difficult to understand elements of the metaphor (Quote 3.1).

One student had difficulty seeing the metaphor of a river as a result of viewing the model from an individualistic western perspective as opposed to the collectivist perspective as suggested by Turpin and Iwama [27]. This is shown in the quote below, where the student converted Kawa Model's concepts into binary westernised ones replacing boulders and driftwood.

“I had to look at my own strengths and weaknesses, so I started to see, ‘Okay, what words do I use to myself to identify… my strengths and weaknesses.'” Kylie

Although some students were challenged by the abstraction of the metaphor, they found that visual resources (Figure 1) received from their practice educator, enabled understanding and the visualisation of the elements and the deep relationships between them. Beyond looking at the templates and engaging in the act of drawing, the students were able to visualise and gauge the influence of elements having an impact on their river flow.

“And also, it is a great way to see visually how much something is impacting you because even though it is not completely accurate, you draw depending on how much it is bothering you, and sometimes, things that you thought would have been a little boulder were actually quite a large boulder compared to the others…” Ava

## 5. Discussion and Implications

The three overarching themes demonstrated intersecting links across the students' experiences of using the Kawa Model in their practice learning in this remote and unfamiliar setting. Self-administration and mutual sharing with a peer of the Kawa Model created opportunities for both mutual understanding and individual self-awareness. This in turn enabled the students to identify personal and professional goals to work on throughout their practice placement. Their increased level of understanding of the metaphor and their drawings of the river was a concrete visual representation of their realistic goal setting and their achievements from one drawing to the next.

The use of the Kawa Model as a reflective tool was found to have elevated and imbued more meaning and value into their reflection processes allowing them to think about their personal and professional development, strengths, and weaknesses (see Quote 1.1.1). In Quote 1.2.1, the students found that the Kawa Model facilitated a noncompartmentalisation of issues, particularly of a temporal nature, and hence, the reflection was seen as being “very effective.”

As the Kawa Model process provided a visual framework that allowed students to initiate self-reflection, they were able to transition from an abstract self-conceptualization to a more tangible self-conceptualization. The repeated visual representation of the Kawa Model created opportunities to scaffold the learning of the students to make sense of their roles in a remote location. These repetitions are supported by Humbert et al.'s [9] findings of the illustrative impact of the Kawa Model in clinical settings. Further, the visual representations of self, in context intersects with Smith's [17] study which found it helped “to organise strengths, weaknesses, assets, liabilities, preferences, and responsibilities concerning each other.”

This visual representation and repetition of the drawings each time a student completed the Kawa Model process enabled them to evaluate their goals through direct comparison to previous drawings by examining the size of the elements of their river and the impact on their river flow. In this way, students were able to identify a large boulder labelled as low confidence and grow smaller as they progressed through the placement demonstrating their improved confidence levels. Mia's quote “It improved my self-awareness in that I had never actually broken it down to think about it” describes the sophisticated nature of the Kawa Model process in that it could be implicitly or explicitly used to enhance self-awareness.

The impact of the iterative visual process facilitated a cognitive reframing of self and is evident in all three themes. Understanding the metaphor was the most difficult aspect of the model for the students, and whilst some students were able to engage better than others, all reported positive outcomes in terms of their learning and professional development. By repeating the Kawa Model process at different times during their remote placement, all the students became aware of the significant personal and professional growth they were experiencing.

Other studies within clinical settings found that the Kawa enhanced team collaboration by facilitating a platform to discuss barriers, facilitators, and goals in the workplace [13, 16, 28]. Aligning with this, students within our study also used the Kawa Model process as a platform to enhance peer collaboration. Engaging in the Kawa Model process provided a space for students to explore their new practice environment and the collaborative skills they would need to participate successfully.

There is limited evidence in the literature of using the Kawa Model with students in rural and remote settings. The students in this study reported using the Kawa Model process to assist them in exploring their sense of self in a remote environment removed from their usual family and learning networks. Using the Kawa Model process in the remote placement created an opportunity for students to self-reflect and develop professional skills to manage their current unfamiliar environments as well as in future placements and careers.

The model guided their thinking beyond the personal, facilitating the integration of their context, environment, culture, and beliefs. This is in keeping with the revised Morris' experiential learning cycle and inclusion of context [24]. Their experience in exploring their sense of self in a rural contextually rich environment echoes the definition of self-awareness by Rasheed et al. [29]. In that, self-awareness occurs on a process continuum, where the person becomes increasingly aware of the personal, intrapersonal, life, and their positionality fostering new behaviours and actions.

Ober and Lape [16, 30] describe enhancing rehabilitation team collaboration through the use of the Kawa Model by “organising, visualising, discussion of goal, barriers, facilitators, and supports.” Another study also describes the use of the Kawa Model as an effective tool for team building [28]. The application of the Kawa Model in this remote setting promoted the students' interpersonal relationships and communication with their peers. Facilitating a novel platform to discuss barriers, facilitators, and goals enhanced their collaboration.

The concept of metacognition has been linked with cognitive and affective processes such as thinking about thinking and learning from learning [28]. This process of continual critical reflection facilitated by the process of completing the Kawa Model process increased students' self-awareness, irrespective of the intended future use of the model. This “metacognitive reasoning” using critical self-reflection is described as “transformative learning” [31, 32]. The students explored their learnings, developing a new sense of themselves. Through this transformative experience of self-reflection and building self-insight, students reported being more motivated and self-confident.

Repetition of the model enhanced the development of professional skills, as student Ella describes “honing-in on smaller areas of your life.” In this student's learning context, these skills included goal planning, communication, and teamwork. Through developing and working towards their goals, students were able to manage the flow of their rivers and thus themselves. Some theorists position themselves as viewing metacognition, self-regulation, and self-regulated learning as being distinct concepts yet sharing self-awareness and regulatory action as a core [33].

Students identified that the repetitive experiential administration of the Kawa Model allowed them to become more confident “by the time I did my third one, I was quite confident, you know, like in making the connections,” reinforcing the value of purposefully designed learning activities that nurture the development of professional confidence. This is supported by Holland et al. [34] who explored community occupational therapists' concept of professional confidence and found that “with experience came professional confidence.”

Understanding the metaphor, revealed a challenge for young adults who are educated within universities that perpetuate or provide curricula informed by Global North perspectives. The metaphor chosen for its universality and ease of application was made difficult by the ontological set of the students. This is visible in the finding that the students initially struggled to fully engage with the model by enhancing their river (life) flow within the context of the various elements of the river. This is an important finding as it has implications for importing the Kawa Model into curricula and for students who have an individualistic and westernised personal and professional positionality.

This study adds new information about how students on practice placement responded to the Kawa Model process as a tool that supported their self-growth in a remote location. Successive Kawa repetitions enabled the students to identify opportunities for personal growth and professional development. The Kawa Model when used in a practice context may be viewed as a vehicle to take students on a transformative learning journey in understanding and self-awareness.

## 6. Limitations

Students administered the Kawa Model with a student peer. Working with a peer may have fostered different reflections as a student may feel reluctant to disclose their thoughts or may have presented a more positive framing of their personal experiences.

In addition, at the commencement of the placement, the students had varying levels of exposure to and experience with the model. All students experienced the same introduction and training in using the model whilst on placement, regardless of their prior knowledge or experience. Those students who had more prior knowledge or experience may have felt more confident in using the model as part of their learning and as a reflective tool.

Students completed the Kawa Model process with varying frequency across their placement journey. The educator encouraged the students to complete their Kawa Model process at the start, midway, and end of the placement, with check-ins in weekly supervision. Outside of these three-time points, completing the Kawa Model process was voluntary, and the frequency of completion was not recorded. Thus, some students might have immersed themselves in the model more fully to promote their learning. During the research interviews, students were not asked to present their own Kawa drawings, and this may have been a missed opportunity to garner important insights into their use.

## 7. Conclusion

This study suggests that the Kawa Model process may be used within the practice context by students, as a self-reflection tool to explore their self-awareness and develop various professional and personal skills such as goal setting and communication. These skills are foundational for the development of entry-level occupational therapists [35]. Despite the challenges some students encountered in understanding the model's metaphor, the iterative nature of the Kawa Model process enabled the development of these skills.

The fact that some students had difficulty understanding the metaphor of the river, offers us an insightful reminder that the metaphor is not fixed and can be modified as described by Ober et al. [13]. Our current habitual use of the Kawa River metaphor should be applied with intention and can be reconfigured with another contextual metaphor for the student.

This research generates further questions regarding the utility of the Kawa Model in occupational therapy student education. We recommend the following (nonexhaustive) list of research questions:

- Explore the Kawa Model process as a self-reflective tool for students' personal development and a self-monitoring tool for skills development earlier in Global North-informed curricula
- Explore students' capacity to transfer learning and use the Kawa Model process in other placement and workplace settings including nonrural settings
- Evaluate the contribution of the Kawa Model to support collaborative peer-assisted learning
- Investigate the role of the educator in facilitating and supporting students to use the Kawa Model
- Further research on the iterative process of using the Kawa Model as part of the supervisory process within rural/remote practice-placement sites
- Compare the use of the Kawa Model with other reflective tools and frameworks to support student development

## Figures and Tables

**Figure 1:** Cross-section of river template. Figure of a cross-section of a river inspired by similar figures in Iwama [4].

**Figure 2:** A composite of a student's Kawa drawing.

**Table 1:** Demographics of sample.

State/territory of university in Australia	Self-declared gender	Previous Kawa experience	Year OT study
Western Australia	Female	Nil	Fourth year
Western Australia	Female	Very brief	Fourth year
Queensland	Female	Yes and prior use	Fourth year
Queensland	Female	Briefly at university	Fourth year
Queensland	Female	Uncertain	Fourth year
Queensland	Female	Briefly at university	Fourth year

**Table 2:** Abridged interview guide.

Topic	Probe questions
Training	(i) What was your experience of working on your own Kawa during training? (ii) How did this influence your understanding of the theory and application of this tool with your clients?

Personal impact	(i) How did this influence your understanding and perception of yourself as a student in training? (ii) How effective was this model in helping you identify your strengths and (ii) weaknesses using the concept of the river? (iii) How did this exercise influence your self-awareness about the flow of your river? (iv) How did you feel the goal planning went and its impact on you? (v) How did the evaluation of your goals work for you? (vi) Describe your experience of using this model and why you would use or not use this model again

Overall	(i) How did you find the application of the Kawa Model in this placement? (ii) And why? (iii) What worked for you? (iv) What did not work? (v) Any suggestions on how to further enhance your understanding of the theory and application of the Kawa model as a tool for assessment and intervention?

**Table 3:** Summary of the interpretative phenomenological analysis (IPA) process implemented.

Steps	IPA process
1	Multiple transcript readings of one case
2	Initial noting of the content of interest (can be very extensive and reflect content, descriptions, linguistic features, or concepts)
3	Developing emergent themes informed by initial notes
4	Grouping emergent themes by bringing together contextual and conceptual ideas and assigning a descriptive label for the theme
5	Analysis of subsequent cases
6	Identifying patterns across cases that generate superordinate themes

**Table 4:** Theme 1: self-awareness.

Theme	Subtheme	Quote
Self-awareness	Self-reflection	1.1.1 “…using it as a tool for reflection, not just doing reflections.” Amelia 1.1.2 “It is definitely good at this point because you get quite caught up in what you need to do next and like the yearly assessments that you have, but it is good to just reflect and to think about your strengths and weaknesses and how you can improve them and move forward and yeah maximise your performance as a student.” Grace
	Self-understanding	1.2 “I noticed things that I thought were not bothering me as something that was still impacting me and how things from my own personal life can impact in my work life…It was very effective in being more aware of myself and my mind and how life is traveling for me and how to improve and what to work on. It even brought up spiritual challenges or strengths in what I believe.” Ava
	Self-evaluation	1.3 “Visual representation of what I am saying is really good to see how much I either believe in myself or I am really doubting myself.” Kylie
	Self-motivation	1.4 “…yeah I think it's good to do on a placement site and I think it is good to do every week. Some weeks you might not invest as much into it and then other weeks you really will and that motivates you to invest even more.” Ava
	Self-confidence/lack thereof	1.5 “By the time I did my third one, I was quite confident, you know, like in making the connections.” Ella

**Table 5:** Theme 2: personal and professional skill development.

Theme	Subthemes	Quote
Personal and professional development	Understanding the model	2.1 “Using it personally first, it does help you consolidate your understanding of the theory underlining it. So, if it was to be used in sequential order, I think definitely using it personally and then with clients” Amelia
	Identify personal growth areas	2.2 “It can help you hone-in because you are now looking at a smaller area of your life, and so, you have to identify all the boulders and that assists to help you in that specific area.” Ella
	Develop goals	2.3 “I'm not very good at goal planning in general, but the Kawa for me, helped me goal plan in what I would kind of be aware of in my practice on the placement, because knowing my weakness, I knew what I wanted to work on through the placement to try and improve myself. So, in that aspect, it was really helpful for planning around that for my goals with the placement.” Kylie

**Table 6:** Theme 3: working with the metaphor.

Theme	Subthemes	Quote
The metaphor	Understanding the metaphor	3.1 “Yeah, I think for me, the river flow is probably the hardest element of the Kawa to understand because it is kind of easier to identify strengths and weaknesses, but you could, if you really honed-in on the model that you did draw, see that there was water still flowing. For me, it was hard to conceptualise what that meant… so that element kind of fell by the wayside because it was not really necessarily understood by myself, yeah.” Amelia
	Visual representation of self	3.2 “And also, it is a great way to see visually how much something is impacting you, because even though it is not completely accurate, you draw depending on how much it is bothering you, and sometimes things that you thought would have been a little boulder were actually quite a large boulder compared to the others…” Ava

## Data Availability

All pertinent data related to this study is included in this article. Raw data shall remain confidential and would not be shared due to ethical reasons.

## Additional Points

*Key Findings*. (i) The Kawa Model may be used as a self-reflection tool for students on remote placement. (ii) Students experienced enhanced self-awareness, self-confidence, self-motivation, communication skills, and professional skills through their engagement with the model. *What the Study Has Added*. This research provides an enhanced understanding of the application and effectiveness of the Kawa Model as a critical reflective tool for occupational therapy students whilst on remote placement.
